The article "Automatic Detection and Segmentation of Ovarian Cancer Using a Multitask Model in Pelvic CT Images" was retracted in 2023. Reasons: suspected computer-generated content; unreliable results or conclusions; concerns about the data; concerns about the results or conclusions.

# Automatic Detection and Segmentation of Ovarian Cancer Using a Multitask Model in Pelvic CT Images

**DOI:** 10.1155/2022/6009107

**Published:** 2022-10-11

**Authors:** Xun Wang, Hanlin Li, Pan Zheng

**Affiliations:** ^1^College of Computer Science and Technology, China University of Petroleum (East China), Qingdao 266580, China; ^2^Department of Accounting and Information Systems, University of Canterbury, Christchurch 8140, New Zealand

## Abstract

Ovarian cancer is one of the most common malignant tumours of female reproductive organs in the world. The pelvic CT scan is a common examination method used for the screening of ovarian cancer, which shows the advantages in safety, efficiency, and providing high-resolution images. Recently, deep learning applications in medical imaging attract more and more attention in the research field of tumour diagnostics. However, due to the limited number of relevant datasets and reliable deep learning models, it remains a challenging problem to detect ovarian tumours on CT images. In this work, we first collected CT images of 223 ovarian cancer patients in the Affiliated Hospital of Qingdao University. A new end-to-end network based on YOLOv5 is proposed, namely, YOLO-OCv2 (ovarian cancer). We improved the previous work YOLO-OC firstly, including balanced mosaic data enhancement and decoupled detection head. Then, based on the detection model, a multitask model is proposed, which can simultaneously complete the detection and segmentation tasks.

## 1. Introduction

Ovarian cancer is called the “no.1 cancer in gynaecology,” and its mortality rate ranks first among gynaecological malignant tumours, which seriously threatens women's lives [1, 2]. Ovarian cancer is difficult to detect at its early stages and progresses rapidly. The lack of effective screening and early diagnosis means that most patients are already at an advanced stage when they are seen and losing the best time for the treatment [3, 4]. In recent years, the number of ovarian cancer patients continues to rise and exhibits a trend of presenting the younger population. Pelvic CT imaging is a common method for diagnosing ovarian cancer [5]. However, ovarian tumours are variable in shape, diverse, and easily adherent to other tissues in a woman's pelvis, which makes the detection of ovarian cancer extremely difficult. It is improbable to avoid misdiagnosis solely based on the diagnostic experience of radiologists. Manual operations are always slow, tedious, and prone to errors. Therefore, there is an urgent need to develop a rapid and accurate automated ovarian cancer detection model [6].

Convolutional neural network (CNN) is a big data-driven model, and since its concept was introduced in 2012, it has been widely used in areas such as image classification, object detection, and image segmentation [7–9]. With the rise of medical big data and deep learning, computer-aided diagnosis system (CADs) develops rapidly [10]. IDTechEx, a well-known British research company, predicts that the market for image-based artificial intelligence medical diagnosis will grow by nearly 10000% by 2040. So far, deep learning has been widely used in the diagnosis of many diseases, such as breast cancer screening, benign and malignant thyroid nodules, and lung cancer detection [11–15].

The article "Automatic Detection and Segmentation of Ovarian Cancer Using a Multitask Model in Pelvic CT Images" was retracted in 2023. Reasons: suspected computer-generated content; unreliable results or conclusions; concerns about the data; concerns about the results or conclusions.

A few research attempts have been using deep learning methods for the diagnosis of ovarian cancer, but most of the research efforts are based on the classification of ovarian cancer after artificial image segmentation. However, it is equally important to identify the location and boundary of the tumour on medical images. Khazendar et al. used SVM for benign and malignant classification on static 2D B-mode ultrasound images of ovarian masses with an average accuracy of 0.77 [16]. Srivastava et al. adopted a fine-tuned VGG16 deep learning network to detect ovarian cysts in ultrasound images, which was able to achieve 92.11% accuracy [17]. Acharya et al. used a fuzzy forest framework in ultrasound images to automatically characterize suspected ovarian tumours with a maximum 80.60 ± 0.5% accuracy, 81.40% sensitivity, and 76.30% specificity [18]. Wu et al. evaluated the performance of four SOTA classification networks: VGG, DenseNet, ResNet, and GoogleNet on a dataset of 988 ultrasound images, with GoogleNet ranking first with an accuracy of 92.50% [19]. In previous work, we proposed an ovarian cancer detection model, YOLO-OC, which achieved an mAP of 73.82% [20].

Compared with ultrasound image, CT image is clearer and has gradually become the first choice for ovarian cancer imaging examination. However, from the research above, it was found that most current CAD systems for ovarian cancer are based on ultrasound images. Thence, this study is dedicated to applying deep learning to the real-time detection of ovarian tumours on CT images.  Figure 1 is an example of this experiment, in which the red dashed border is the ground truth marked by a professional radiologist. It can be seen from Figure 1 that the tumour has no fixed shape and the boundary with normal tissue is not clear, which requires the proposed model to have a strong feature extraction ability.

The proposed model YOLO-OCv2 is based on YOLOv5. Our first attempt at the problem developed the network model YOLO-OC which is YOLOv3 based [20]. YOLO-OC uses deformable convolution to capture the geometric deformation in space. In YOLO-OCv2, three modules are designed and developed to improve the performance of the model so that it can detect ovarian cancer more accurately on pelvic CT images. Furthermore, we introduce the segmentation head at the appropriate location and explore the internal module composition of the segmentation head.

1. In view of the problem of few samples and unbalanced types of ovarian cancer CT datasets, we add the principle of the softmax formula to the sampling process of mosaic enhancement to balance the probability of each type of sample being selected. The second improvement is to replace the SE attention mechanism [21] used by YOLO-OC with the coordinate attention mechanism [22]. Finally, the output of the model abandons the coupled detection head that the original YOLO model has always used. We design a decoupled head to output classification, regression, and confidence separately, and any branch can be optimized separately
2. In the YOLO-OCv2 model, this paper proposes a multitask model, which can simultaneously complete the task of ovarian tumour object detection and semantic segmentation, and the addition of the segmentation head will not have side effects on the detection effect

The rest of the paper is organized as follows. In Section 2, we briefly introduced the current mainstream object detection networks and multitask models and sorted out the development of the YOLO series of detectors. In Section 3, we introduced the dataset used in the experiment and the detailed architecture of the proposed model. In Section 4, we presented an extensive evaluation of the results of the proposed model. In Section 5, we summarized the entire paper and discussed future prospects.

The article "Automatic Detection and Segmentation of Ovarian Cancer Using a Multitask Model in Pelvic CT Images" was retracted in 2023. Reasons: suspected computer-generated content; unreliable results or conclusions; concerns about the data; concerns about the results or conclusions.

## 2. Related Work

Object detection, one of the fundamental problems of computer vision, is the basis for many other computer vision tasks, such as instance segmentation and object tracking. The problems solved by the object detection algorithms are what objects they are and the whereabouts of the objects. Multitask learning is aimed at learning better semantic representations by exploiting shared feature information among multiple tasks, especially CNN-based multitask learning methods which can achieve convolutional sharing of network structures.

### 2.1. Object Detection

The object detection model is divided into a one-stage detector and a two-stage detector. YOLO is the most commonly used one-stage detector in the research field. We will explain the development of the YOLO model in detail in Section 2.2. RefineDet is a combination of the single-shot multibox detector (SSD) algorithm, region proposal network (RPN), and feature pyramid network (FPN), which can improve the detection effect while maintaining the efficiency of the SSD algorithm [23]. EfficientDet is a series of object detection algorithms, including a total of eight algorithms from D0 to D7. It proposes a weighted bidirectional feature pyramid network (BiFPN) and uniformly scales the resolution, depth, width, and feature fusion network of all backbones [24]. Furthermore, anchor-free detectors have attracted more and more attention in recent years, which do not need a prior anchor to match the object. Its representatives include Fully Convolutional One Stage Detector (FCOS), ExtremeNet, and CornerNet, whose performance can already compete with SOTA anchor-based detectors [25–27]. A recent YOLOv5 application is to detent underwater maritime objects [28], which has a good identification result in very short time interval.

The article "Automatic Detection and Segmentation of Ovarian Cancer Using a Multitask Model in Pelvic CT Images" was retracted in 2023. Reasons: suspected computer-generated content; unreliable results or conclusions; concerns about the data; concerns about the results or conclusions.

### 2.2. YOLO Object Detection Model

So far, YOLO series detectors have been developed to YOLOv5. They are widely used in practice due to their high efficiency and fast speed. The core idea of YOLO is to use the entire image as the input of the network and directly regress the position and category of the bounding box in the output layer. YOLOv1–YOLOv3 are all developed and maintained by Redmon et al. [29–31]. YOLOv4 was proposed by Alexey AB and it builds on YOLOv3 with many SOTA bag-of-freebie and bag-of-special tricks [32]. The bag of freebies refers to tricks that can increase model accuracy without increasing the amount of inference calculations, including data augmentation and GIoU loss. Besides, bag of specials refers to some plugin modules (such as feature enhancement models or some postprocessing), which increase the amount of calculations a little but can effectively increase the accuracy of object detection. YOLOv5 is a version implemented by Ultralytics based on PyTorch. In addition to adding many tricks, it also scales the model for network design.

### 2.3. Multitask Model

The general feature information of the backbone provides a theoretical basis for the construction of multitask models. Based on this, many excellent multitask models have been born in the field of computer vision. Mask RCNN adds a Mask branch on the basis of Faster R-CNN to predict the Mask on the region of interest and achieves good results in object detection and instance segmentation tasks [33]. Multinet is a research achievement in the field of real-time automatic driving. The three subtasks share a VGG16 encoder backbone, which can realize end-to-end training and complete three independent scene perception subtasks: scene classification, object detection, and driving area segmentation in only 98.10 milliseconds [34].

The article "Automatic Detection and Segmentation of Ovarian Cancer Using a Multitask Model in Pelvic CT Images" was retracted in 2023. Reasons: suspected computer-generated content; unreliable results or conclusions; concerns about the data; concerns about the results or conclusions.

## 3. Ovarian Cancer Detection Model

Before we describe the proposed model, it is necessary to mention the motivation for it. As described in Introduction, to accurately detect ovarian tumours on CT images, it is necessary to improve the model's ability to extract key features. Therefore, we introduce the coordinate attention module and decoupling head in the baseline.  Figure 2 shows the module details of our proposed model, which follows the multiscale detection of the YOLO detector.

### 3.1. Overall Network Structure

YOLO has always used the lightweight Darknet as the backbone to ensure the forward inference speed, but its feature extraction ability is slightly insufficient for medical image detection tasks. The YOLO-OCv2 model proposed in this paper improves the original YOLO model based on a specific ovarian cancer detection task. The image is histogram equalized before being input to the model. The input of batch size dimension is constructed by the balanced mosaic enhancement module.

The convolution used for feature extraction in backbone C5 is replaced with deformable convolution [35], enhancing the geometric modelling capabilities of the model. The feature map extracted by the backbone first enters the Class Attention (CA) layer and then enters the spatial pyramid pooling (SPP) layer. The feature fusion layer adopts PANet [36]. Compared with FPN [37], it has one more feature fusion process from bottom to top. Finally, Path Aggregation Network (PANet) outputs feature maps of different sizes into the decoupling head.

### 3.2. Balanced Mosaic Module

Mosaic enhancement is a simple and effective way of data enhancement, which is an improvement to CutMix enhancement. The advantage of mosaic enhancement is that it enriches the background information of the object to be inspected and the number of small objects and during batch normalization.  Figure 3 shows that the mean and variance of the four images are calculated at once, which greatly improves the robustness of the model.

Softmax is often used in the last layer of machine learning models to output classification probabilities. Different from Hardmax's enlargement strategy, the key of softmax is “soft,” which can shorten the distance between nodes. In addition, with the feature that the sum of softmax output results is 1, we combine it with mosaic enhancement. Firstly, count the number of objects in each category, then get the probability of each category being selected in the original mosaic enhancement, take the probability value as the input node of softmax, namely, *V*_*i*_ in the formula, and reoutput the probability of each category being selected.

(1) $$\begin{array}{c} S_{i}=\frac{e^{V_{i}}}{\sum_{j}e^{V_{i}}}. \end{array}$$

The article "Automatic Detection and Segmentation of Ovarian Cancer Using a Multitask Model in Pelvic CT Images" was retracted in 2023. Reasons: suspected computer-generated content; unreliable results or conclusions; concerns about the data; concerns about the results or conclusions.

### 3.3. Coordinate Attention

In essence, the attention mechanism in deep learning is similar to the selection and filtering mechanism of the human eye. The key is to select the most important feature information for the current task from a large number of features. Aiming at the problem of unclear boundaries and difficult identification of ovarian tumours, this paper explores a new attention mechanism: coordinate attention [22].

Unlike SE block, which uses two-dimensional global pooling to convert input feature maps into a single feature tensor, CoordAttention (Figure 4) decouples channel attention into one-dimensional feature encoding processes in both horizontal (*X*) and vertical (*Y*) directions. The advantage of this design is that while capturing long-term dependencies in one spatial direction, it can accurately retain the positional information in another spatial direction, making up for the lack of positional attention information in SE blocks. These output feature maps are then separately encoded to form a pair of orientation-aware and position-sensitive feature maps, which combined with the input feature maps can enhance the representation of ROI objects.

### 3.4. Decoupling Head

The role of the detection head in the detection model is to convert the output of the model into human-defined semantics, such as category and confidence. The YOLO model has always used a coupled head, that is, all feature maps are output through a final calculation in one step, and the feature maps of different channels represent different semantic information. The decoupling head is a standard component of detection models such as RetinaNet and FCOS. In the work of YOLOX, it was found that the original YOLO detection head lacks the expressive ability [38]. After switching to the decoupling head, the network not only improves its peak performance but also significantly accelerates its convergence speed, which proves that the coupling head used by YOLO series models is unreasonable.

We also designed the coupling head in YOLO-OCv2, as shown in Figure 5. Decoupling the detection head for multibranch output will undoubtedly increase the complexity of the model. Therefore, we first use convolution to reduce the dimension of the features, compress the number of channels, and then output through the classification and regression branches, respectively. The regression branch (box) and the confidence branch (obj) share a set of convolution kernels. Another branch (cls) is the class of each bounding box. Finally, all feature maps are superimposed in the channel dimension, and the final decoding process of the model remains unchanged.

The article "Automatic Detection and Segmentation of Ovarian Cancer Using a Multitask Model in Pelvic CT Images" was retracted in 2023. Reasons: suspected computer-generated content; unreliable results or conclusions; concerns about the data; concerns about the results or conclusions.

## 4. Multitask Model Based on YOLO-OC

### 4.1. Multitasking Model Structure

The multitask model adds a segmentation head based on YOLO-OCv2, and the two subtasks share the encoder weights of YOLO-OCv2. The image is first processed by adaptive histogram equalization and then enhanced by the balanced mosaic. The overall structure of the model is shown in Figure 6, and the encoder part is consistent with the detection model above. The selection of the segmentation head position will be shown in detail later. In addition, we also discussed the impact of the ASPP module proposed by Deeplabv2 [39].

### 4.2. Segmentation Head Position

There are three options for the location of the segmentation head. One is to connect the segmentation head at the last layer of the FPN as shown in Figure 7(a). Another scheme is shown in Figure 7(b); the segmentation head is connected after the maximum resolution feature map in the path from the bottom to the top of PANet. There is little difference between the two methods, and only one scale feature map is used for upsampling. This design only uses the top-down feature fusion in PANet, while the semantic fusion function of the other path is not used. In order to maximize the use of semantic features, we also designed the third scheme.

The third scheme is shown in Figure 8, in which the minimum resolution feature map and the medium resolution feature map output by PANet are stacked with the large resolution feature map through upsampling. The feature map fused with multilayer semantic information finally enters the designed segmentation head for the segmentation task, and the position of the decoupling head used for detection remains unchanged.

### 4.3. The Composition of Segmentation Head

The composition of the segmentation head is shown in Figure 9. The feature map first goes through a convolution layer to reduce the dimension. Because the ASPP module requires a large amount of computation, reducing the number of feature channels can effectively reduce the amount of computation and parameters. Then, the feature map enters an ASPP module to extract the semantic information of different receptive fields, which fully proves its effectiveness in the Deeplab model. The output features learn the channel weights in the SE channel attention module and finally upsample to the original image size to output pixel-level classification.

As shown in Figure 10, different from the conventional spatial pyramid pooling (SPP), atrous spatial pyramid pooling (ASPP) arranges whole convolutions with different expansion rates in parallel for feature extraction and plays the role of capturing feature context using multiple proportions. In the experimental results of Deeplabv2, this module can bring great performance improvement. Therefore, ASPP is often used in some subsequent detection and segmentation models.

The article "Automatic Detection and Segmentation of Ovarian Cancer Using a Multitask Model in Pelvic CT Images" was retracted in 2023. Reasons: suspected computer-generated content; unreliable results or conclusions; concerns about the data; concerns about the results or conclusions.

## 5. Experiments

### 5.1. Datasets and Evaluation Metrics

The pelvic CT datasets used in this study are from the Affiliated Hospital of Qingdao University, China, which is a comprehensive grade 3A hospital. After filtering out some unclear data, we obtained a total of approximately 5100 CT images of 223 patients. Then, we anonymised the image data to remove the sensitive information of the patients, hence protecting the privacy of the individuals. According to the manual annotation of professional radiologists in Figure 1, we used the annotation tool to establish the ground truth of the dataset. The number of samples of each type in the ovarian cancer dataset is shown in Table 1, and the number of samples of serous cystadenoma cancer is much larger than that of other types.

In order to verify the performance of our proposed model, we used 6 indicators to quantitatively evaluate our model, which include precision, recall, *F*1 score, mean average precision (mAP), mean pixel accuracy (MPA), and mean intersection over union (MIoU). mAP@0.5 corresponds to the average detection precision of the IOU threshold of 0.5. By default, mAP refers to mAP@[0.5,0.95], which is the average mAP at different IOU thresholds (from 0.5 to 0.95, with a step size of 0.05).

(2) $$\begin{array}{c} \text{precision}=\frac{\text{TP}}{\text{TP}+\text{FP}},\\ \text{recall}=\frac{\text{TP}}{\text{TP}+\text{FN}},\\ F1=\frac{2*P*R}{P+R},\\ \text{mAP}=\frac{1}{C}\overset{C}{\underset{j}{\sum }}{AP}_{j},\\ \text{MPA}=\frac{1}{k+1}\overset{k}{\underset{i=0}{\sum }}\frac{p_{ii}}{\sum_{j=0}^{k}p_{ij}},\\ \text{MIoU}=\frac{1}{k+1}\overset{k}{\underset{i=0}{\sum }}\frac{p_{ii}}{\sum_{j=0}^{k}p_{ij}+\sum_{j=0}^{k}p_{ji}-p_{ii}}. \end{array}$$

### 5.2. Implementation Details

All experiments in this study were run on a host with NVIDIA GeForce RTX 2080 Ti GPU and 6-core Intel CPU. The skeleton of the proposed model in this paper was built by PyTorch 1.7. In the model training phase, we applied an initial learning rate of 0.01, which decreased as the training batch increased. In addition, we adopted stochastic gradient descent (SGD) to optimize our proposed network, where momentum and weight decay were set to 0.937 and 0.0005, respectively. Limited by the GPU computing power, the batch size was set to 8, and all models were trained for 100 epochs.

### 5.3. Ablation Experiment

The first improved module proposed in this study is the balanced mosaic enhancement module, which can balance the number of samples according to the reconstructed prior probability during mosaic splicing, thereby effectively alleviating the problem of class imbalance. As shown in Table 2, the original mosaic enhancement has a great improvement over the original image input, but still does not solve the problem of class imbalance. After adding balanced mosaic enhancement, the AP of serous cystadenoma carcinoma was only reduced by 0.10%, while the accuracy of the other four categories was improved, and the overall accuracy was improved well. The results show that this module can effectively improve the problem of class imbalance.

The article "Automatic Detection and Segmentation of Ovarian Cancer Using a Multitask Model in Pelvic CT Images" was retracted in 2023. Reasons: suspected computer-generated content; unreliable results or conclusions; concerns about the data; concerns about the results or conclusions.

Table 3 intuitively shows the model performance improvement brought by each component in YOLO-OCv2, where DCN is deformable convolution and CA is coordinate attention mechanism. While the decoupling head only increases a limited amount of parameters, it effectively improves the detection accuracy. By combining these four strategies, we can continuously improve the mAP value of the detection network without performance degradation due to module conflicts. Compared with the original YOLO, YOLO-OCv2 finally improves mAP by 3.31%.

Table 4 shows the impact of the three positions of the segmentation head on the performance of the model. The positions of scheme 2 and scheme 1 are similar, and the low-resolution feature maps are not fused twice. Compared with scheme 1 and scheme 2, scheme 3 has an increase of 1.69% and 1.66% in MIoU and an increase of 1.22% and 1.15% in MPA, respectively. Experiments show that the fusion of secondary semantics helps the model to learn more fine-grained semantic information.

The results of the ablation experiments in the segmentation head are shown in Table 5. We have tried three attention mechanisms, namely, SE, CBAM, and CA. CBAM is a dual attention mechanism like CA [40], including spatial attention and channel attention. The experimental results show that the ASPP module has a great impact on the performance of the model. After adding ASPP, the MIoU and MPA of the multitask model are increased by 1.52% and 1.3%, respectively. In terms of attention module, SE can improve MIoU by 0.35% and MPA by 0.27%, while the other two more complex attention mechanisms are not as good as simple channel attention. The possible reason is that the previous ASPP module has been fully learned with the location information.

### 5.4. Comprehensive Comparison

Table 6 shows the performance of YOLO-OCv2 and several common object detection networks (Faster R-CNN, SSD, and RetinaNet) on our test set. The pretrained models used to initialize the weights of each model are all trained on the COCO dataset.

Four contemporary methods used to solve relevant problems are selected to benchmark with our methods, namely, Faster R-CNN (region-based convolutional neural network), SSD (single-shot detector), RetinaNet, and YOLOv5. These four methods and algorithms were chosen as they are among the most popular and influential deep learning methods in feature detection. The experimental results show that the proposed YOLO-OCv2 network has the best detection performance of ovarian cancer with the datasets.

The article "Automatic Detection and Segmentation of Ovarian Cancer Using a Multitask Model in Pelvic CT Images" was retracted in 2023. Reasons: suspected computer-generated content; unreliable results or conclusions; concerns about the data; concerns about the results or conclusions.

The qualitative detection results of YOLO-OC are shown in Figure 11. The method can accurately locate and classify different types of ovarian tumours. It indicates that the model proposed in this paper has the potential to assist radiologists in accurately diagnosing the tumours.

The segmentation results are shown in Table 7. For the ovarian cancer pelvic CT image dataset, the evaluation indicators of our proposed multitask model are higher than those of the other semantic segmentation networks. Similar to the experimental conclusion of Mask RCNN, the detection performance of the multitask model did not drop but increased a little compared to the original YOLO-OCv2 model, indicating that the backpropagation of the segmentation head helps to optimize the features and improve the detection performance.

Figure 12 shows the input original image, ground truth, and the output of the multitask model from left to right. It can be seen from the figure that the multitask model has a good segmentation effect and also has a good segmentation effect on irregular boundary areas.

## 6. Conclusions

In order to solve the practical clinical problems, this study investigated the research status of ovarian cancer medical image detection and recognition and elaborated on the research significance of this task. Drawing on the excellent research results in the field of computer vision, we propose a model YOLO-OC for ovarian cancer CT image detection, which can accurately locate and identify tumour lesions. Finally, based on the YOLO-OC model, a segmentation head for semantic segmentation is added to achieve end-to-end detection and segmentation tasks at the same time.

The results generated by our algorithm are convincing and with excellent accuracy by comparing with the state-of-the-art algorithms; however, there are a few limitations and places for improvement of our methods. The internal structure of the network is complex which directly imposes a high level of computational cost. In the future, the proposed method can be streamlined and deployed for real-time applications and systems in hospital settings. The proposed method is semantic segmentation. The objective is to identify and segment the ovarian tumour out of the surrounding healthy organisms. Technically, YOLOv5 can be used for instance segmentation. It is with the higher priority of the study to achieve our primary objective. Instance segmentation may provide some value-added characteristics, e.g., to identify individual nodules of a big block of tumour organism. It could be one of the future directions of this study.

The article "Automatic Detection and Segmentation of Ovarian Cancer Using a Multitask Model in Pelvic CT Images" was retracted in 2023. Reasons: suspected computer-generated content; unreliable results or conclusions; concerns about the data; concerns about the results or conclusions.

## Figures and Tables

**Figure 1:** This experiment classified ovarian tumours into five categories: (a) serous cystadenoma carcinoma; (b) clear cell carcinoma; (c) mucinous cystadenoma carcinoma; (d) endometrioid carcinoma; (e) others.

**Figure 2:** The overall design of the YOLO-OCv2 network structure.

**Figure 3:** Mosaic augmentation's splicing schematic.

**Figure 4:** The process of coordinate attention (CA) block.

**Figure 5:** Decoupling head structure in YOLO-OCv2.

**Figure 6:** The overall architecture of the multitasking model in YOLO-OCv2.

**Figure 7:** Segmentation head position selection.

**Figure 8:** The third scheme of segmentation head position.

**Figure 9:** The internal module composition of the segmentation head.

**Figure 10:** ASPP internal module composition.

**Figure 11:** Examples of YOLO-OCv2 detection effects.

**Figure 12:** (a) Original image; (b) ground truth; (c) final output.

**Table 1:** The number of data used for training and testing.

Category	Training	Testing
Endometrioid	347	62
Clear cell	375	66
Mucinous	390	68
Serous	2901	513
Others	367	64

**Table 2:** Improved mosaic augmentation vs. before improvement.

Category	Endometrioid	Clear cell	Mucinous	Serous	Others	mAP (all)
No mosaic	70.52%	70.28%	69.84%	75.09%	68.97%	70.94%
Mosaic	71.06%	71.12%	70.92%	75.45%	69.15%	71.54%
Balanced mosaic	71.66%	71.87%	71.59%	75.35%	69.83%	72.06%

**Table 3:** Ablation study results of the YOLO-OC model.

Backbone	Balanced mosaic	DCN	CA	Decoupling head	mAP@[0.5,0.95]
CSPDarknet53	√				72.06%
CSPDarknet53	√	√			73.24%
CSPDarknet53	√	√	√		73.77%
CSPDarknet53	√	√	√	√	74.85%

**Table 4:** Performance differences for different segmentation head positions.

SegHead position	MIoU	MPA
Case 1	87.94	91.49
Case 2	87.97	91.56
Case 3	**89.63**	**92.71**

**Table 5:** Comparison of results from ablation studies of segmentation heads.

Model				MIoU (%)	MPA (%)
ASPP	SE	CBAM	CA		
				87.76	91.14
**√**				89.28	92.44
**√**	**√**			**89.63**	**92.71**
**√**		**√**		89.51	92.59
**√**			**√**	89.60	92.63

**Table 6:** Performance comparison of YOLO-OC with other classical models.

Model	mAP@0.5	mAP@0.75	mAP@[0.5,0.95]	*F*1 score	FPS
Faster R-CNN	89.64%	82.84%	71.56%	85.94%	0.8
SSD	88.30%	79.32%	68.79%	85.33%	5.2
RetinaNet	90.81%	83.40%	71.97%	88.75%	4.3
YOLOv5	87.96%	82.25%	71.54%	87.83%	10.3
YOLO-OCv2	92.21%	85.66%	74.85%	89.85%	9.4

The article "Automatic Detection and Segmentation of Ovarian Cancer Using a Multitask Model in Pelvic CT Images" was retracted in 2023. Reasons: suspected computer-generated content; unreliable results or conclusions; concerns about the data; concerns about the results or conclusions.

**Table 7:** Performance of multitask models and other classic models on ovarian cancer datasets.

Model	Ovarian cancer dataset		
	MIoU	MPA	mAP@0.5
FCN	80.53	85.07	
SegNet	81.88	85.26	
U-Net	85.97	88.19	
Deeplabv2	88.75	90.43	
Multitask model	**89.63**	**92.71**	**92.37**

## Data Availability

Data is available upon request and consent of relevant hospitals.
